The article "Large-Scale Textual Datasets and Deep Learning for the Prediction of Depressed Symptoms" was retracted in 2023. Reasons: signs of a paper mill; suspected computer-generated content; unreliable results or conclusions; lack of ethics approval or compliance.

# Large-Scale Textual Datasets and Deep Learning for the Prediction of Depressed Symptoms

**DOI:** 10.1155/2022/5731532

**Published:** 2022-04-12

**Authors:** Sudeshna Chakraborty, Hussain Falih Mahdi, Mohammed Hasan Ali Al-Abyadh, Kumud Pant, Aditi Sharma, Fardin Ahmadi

**Affiliations:** ^1^Computer Science & Engineering, Lloyd Institute of Engineering and Technology, Greater Noida, India; ^2^Computer Engineering Department, University of Diyala, Iraq; ^3^Prince Sattam Bin Abdulaziz University Alkharj Saudi Arabia, College of Education- Thamar University, Thamar, Yemen; ^4^Department of Biotechnology, Graphic Era Deemed to Be University, Dehradun, Uttarakhand, India; ^5^Computer Science Engineering & Information Technology, Institute of Engineering & Technology, Lucknow, Uttar Pradesh, India; ^6^Rana University, Kabul, Afghanistan

## Abstract

Millions of people worldwide suffer from depression. Assessing, treating, and preventing recurrence requires early detection of depressive symptoms as depression-related datasets expand and machine learning improves, intelligent approaches to detect depression in written material may emerge. This study provides an effective method for identifying texts describing self-perceived depressive symptoms by using long short-term memory (LSTM) based recurrent neural networks (RNN). On a huge dataset of a suicide and depression detection dataset taken from Kaggle with 233337 datasets, this information channel featured text-based teen questions. Then, using a one-hot technique, medical and psychiatric practitioners extract strong features from probably depressed symptoms. The characteristics outperform the usual techniques, which rely on word frequencies rather than symptoms to explain the underlying events in text messages. Depression symptoms can be distinguished from nondepression signals by using a deep learning system (nondepression posts). Eventually, depression is predicted by the RNN. In the suggested technique, the frequency of depressive symptoms outweighs their specificity. With correct annotations and symptom-based feature extraction, the method may be applied to different depression datasets. Because of this, chatbots and depression prediction can work together.

## 1. Introduction

Depression is a regular occurrence in the workplace, school, and home stress can all contribute to depression [1]. Adults are affected by adolescent depression; approximately 0.8 million individuals commit suicide each year [2, 3]. Mental illnesses account for five of the top 10 debilitating conditions, with depression being the most frequent [4]. As a result, depression is a serious illness. More than half of all people have mild depression [5]. Adults in their forties and fifties are particularly vulnerable. When depression is recognized early, it is easier to treat [6–10]. However, identifying depression symptoms requires time and effort. To predict mental illness, physician interviews and hospital or agency questionnaire surveys [11] are now employed. One-on-one surveys are used in this method.

Instead of interviews or questionnaires, spontaneous writings submitted by users can be used to forecast depression. Clinical psychology has looked into the link between a language user (speaker or writer) and their text [12]. Havigerova et al. found that trip-related informal language might predict depression in recent research [12]. As a result, electronic records and data are becoming more vital in health care. The application of recent breakthroughs in natural language processing and artificial intelligence to detect depressive symptoms in informal writing is promising for artificial intelligence (AI). Linguistics and computing are used to help computers interpret text. The goal in this scenario is to assign negative or positive polarity to opinions, ideas, and concepts. Automated text analysis in conversations or blog postings can detect depressive symptoms [13–18]. However, there is still a lot to learn about reading letters for melancholy. It is difficult to write about serious depression. Depression symptoms are difficult to diagnose with a single statement. Our automated detection method, we feel, can make a significant scientific contribution. As a result, the present study uses artificial intelligence to detect depressive signs in the text.

Linear discriminant analysis (LDA) is an excellent method for visualizing discriminant data [19–22]. It operates by grouping comparable samples together. Its goal is to improve between-class scatter while lowering within-class dispersion. Facial expression recognition and human activity recognition are examples of real-world LDA applications. The dimensionality of class data is reduced using LDA.

Deep neural networks have lately aided in pattern recognition and AI research [23–34]. It does, however, have two big flaws. The first fault is that it is very tight. Data modeling takes a long time. Restricted Boltzmann machines (RBMs) were used to speed up training in the early days of deep learning. A better instrument for discriminating than others. Convolution neural network (CNN) extracts and trains its data. An abstract feature hierarchy may be created using convolution [24]. Instead of analyzing time-series data, CNNs are employed for image and video analysis. In the examination of sequential data and patterns, RNNs outperform CNNs [30]. For high-dimensional and time-correlated input, RNNs employ LSTM to overcome the problem of vanishing gradients. An LSTM-based RNN is therefore employed in this work to mimic emotional content in text data.

Human physical and mental functions have been extensively studied using machine learning [35–41]. Industry stakeholders are requesting more openness when machine learning algorithms are used to provide crucial forecasts [42]. The major danger is creating and implementing bad AI judgments. The list goes on. Precision medicine practitioners, for example, require more than mere machine learning predictions to support their diagnosis. Other professions, such as medicine, may have similar requirements. In rare cases, this may result in system rejection. Recent research emphasizes the necessity for explainable AI to build trust in machine learning results. Local interpretable model-agnostic explanations (lime), Shapley additive explanation (SHAP), and layerwise relevance propagation are only a few of the modern explanation algorithms that may be used nowadays. Layerwise relevance propagation (LRP). As a result, lime is small and focused on offering quick, posthoc explanations. As a result, when the model is completed, this study will make use of lime to determine why (importance of the attributes). The goal of this project is to identify depressive symptoms in text for a smart chatbot application. Text queries are processed by the server using feature extraction and deep learning. The findings may lead to additional suggestions from the server. RNN features are developed from all user text input throughout the training phase.

Based on the test results, the trained model determines if the user is sad. To compare proposed features to existing features, LDA is utilized. Finally, we use a widely used method to produce posthoc, local, and understandable machine learning explanations. Here is how the paper makes a difference:

Medical and psychiatric professionals point out certain characteristics that might indicate depression. To imitate emotions, it employs LSTM, attention, and thick layers.  Section 2 shows information gathering and analysis.  Section 3 depicts methodology. Sections 4 and 5 explain results and conclusion, respectively.

## 2. Information Gathering and Analysis

Recognizing mental health disorders necessitates the gathering of data. Social media data, such as Facebook status updates, is insufficient. [43]. Use of the massive text-based dataset on the ung.no public information website. On ung.no, young people can anonymously ask questions in Norwegian. Answers and counseling are provided by professionals (doctors, psychologists, nurses, and so on). These are made available to the public via the Internet. Teenagers define and categorize their postings on ung.no. The topic for this week was “emotions and mental health.” They are usually short, but they describe the mental state, symptoms, and behavior. To begin with, some of the writings depict depression that has been medically diagnosed. Many texts examine the history and symptoms of depression, either rejecting or confirming the diagnosis. They appear to be an expression of self-perceived sadness. Clinical diagnoses are mirrored in self-perceived mental states [44–46]. There are a few words that tell tales and portray emotions without using the word “sad.”

It is thought to be depressive symptoms. One of the data categories is depression. The signs of depression were then validated by a competent general practitioner. Melancholy is determined by analyzing a set of phrases and words. The accusations were corroborated by a doctor. In the appendix, you will see possible remarks and/or terms that unhappy kids could use in their searches. To get features for each message, use phrases and words. Look at Table 1 to learn about depression in English. There were 277,552 posts in all, including depressing messages. From that dataset, we used 11,807 and 21,470 postings in our two investigations. Text features are used as binary patterns in a depression prediction machine learning model. The following list of stemmed terms demonstrates the breadth of terminology related to depression [47].  Table 2 displays the snapshot of the dataset taken for the analysis purpose.

## 3. Methodology

The proposed methodology is discussed in the section, here preprocessing is the first part of the method and then modeling and the proposed model are given.

### 3.1. Preprocessing

The survey questions are put in rows in the dataset, and the survey participants are grouped into columns, resulting in distinct health domain tables. Because the tables are not all organized in the same way, preprocessing is required to categorize the data. For our research, we will only use one-third of the dataset: the survey questions. To eliminate duplicates and make it more computer-readable, the data was cleaned and modified. The data formats were chosen to allow for comparisons and contrasts between the datasets. To establish a uniform scale across all of the questions, normalization was also necessary. When data is prepared to utilize psychological domain information from functional diagnostic criteria, the data structure is reconstructed. All tables should be reconstructed using just six functional categories of depression diagnostic criteria. It makes no difference whether there are more or fewer questions because the participants are all the same. The six tables may be consolidated into one because they all have the same row index. When each table is instantly seen, it generates a new dataset with participants as instances and questions as features.

### 3.2. Classification by Modeling

An ensemble classification approach is used to build the model. Many classification algorithms are used simultaneously using Independent Ensemble Methodology (IEM). The model employs the support vector machine, artificial neural network, K-nearest neighbor (KNN), and decision tree algorithms. In a single training run, each composite classifier is trained on the same piece of training data. A k-fold cross-validation approach is utilized as a part of the assessment process. The ensemble classifier is built by merging the results of all the composite classifiers into a single prediction. An ensemble classification technique employs many independent classifiers to improve prediction accuracy.

An ensemble method, on average, outperforms a single algorithm in terms of prediction performance. The advantages of performance:

- By averaging numerous alternative hypotheses, an incorrect hypothesis is avoided from being chosen.
- Combining several learning ensemble approaches reduces the possibility of reaching a local minimum, which saves time and money.
- Using numerous models and diverse representations, we were able to improve the data fit and extend the search area.

The ensemble approach simulates human behavior by looking at a variety of choices. When we compare our preprocessed data to other baseline models, we may conclude that the ensemble strategy for this experiment is a superior technology.

An ensemble model is exemplified by this. The accuracy of predictions is anticipated to increase if all four techniques are used together. Training each of the ensemble's various submodels is required to broaden the scope of the ensemble classifier. To combine the outputs from all of the initial classifiers in our model, we employ a weighted ensemble technique. A weighted ensemble strategy is incredibly broad due to the same outputs of each base classifier. The weights of classifiers are determined by their accuracy on a validation set.

It is fantastic to use a machine learning model to decode time-series data. Therefore, RNNs are employed. [22] RNNs are commonly employed to represent time-sequenced data. In RNNs, previous and present states are linked through recurrent connections. Neural networks rely heavily on memory. A vanishing gradient problem or a processing limit is a common problem for RNN algorithms. The text feature extraction and the suggested model are listed as follows: Figure 1 depicts the sample post with words belonging to depression and nondepression category.

## 4. Experimental Results

We used data from Kaggle.com. There are depression-related texts included in the collection. Some of the communications were annotated by medical and psychiatric professionals. Testing was conducted on a 32 GB RAM, Windows 10, and the TensorFlow 2.4.1 deep learning tool with an Intel (*R*) Core (TM) 7700HQ CPU operating at 2.8 GHz and 2.81 GHz.

### 4.1. Dataset and Experiments

For the first dataset and trials, there were 11,807 messages in total, with 1820 of those identified as depression texts (detailed descriptions of depression symptoms) and 9987 of those classified as nondepression texts (not describing symptoms of depression). These tables show the tenfold classification reports used in most of the training and testing datasets.

During tenfold training, the accuracy and loss are shown in Tables 3–5. Fold training looks to be going well, except for a slight tweak. This approach's confusion matrix is depicted in Figures 2 and 3 for folds 1 and 2. The suggested features outperform one-hot and LSTM with mean recall rates of 0.98 and 0.99 for depression and nondepression, respectively. When comparing precision levels, the precision-recall curve illustrates the trade-off between accuracy and recall. A large area under the curve indicates that the person has strong recall and accuracy. Because high accuracy implies low false positives, and strong recall implies low false negatives, high accuracy implies low false positives.

Accuracy at the 0.99 level indicates that the method is long-lasting.

Figure 4 shows the machine learning model's overall probability. In most ways, a three-dimensional scatter plot is comparable to a two-dimensional scatter plot. Scatter plots are often used to illustrate the relationship between two numbers. Positive or negative, strong or weak, linear or nonlinear relationships between two variables may be depicted in a number of ways. Additionally, scatter plots may aid you in detecting other patterns in the data.

Emotional states' one-hot characteristics, TF-IDF characteristics, and LDA's projected strong characteristics are depicted in three-dimensional renderings in Figures 5–8 in this section.

The mean accuracy (percentage) and forecast accuracy (percentage) for different approaches to all participants are also presented in Table 6.

One of the study's possible benefits is assisting users who show indicators of depression but have not yet been officially diagnosed. In general, the earlier patients get help for depression, the better their outcomes and costs. An intrusive marketing tactic used by mental health organizations to target potential customers based on their web behavior may be deemed intrusive. People are skeptical of this strategy based on preliminary findings. Explainability and interpretability are important factors in overcoming the barrier of using social media data for mental health prediction models.

## 5. Conclusion

This study's goal was to develop a multimodal human depression prediction strategy using RNN deep learning and robust depression symptom features. First, text data from suicide datasets for young users is first used. An on-hot approach is then used after extracting words from phrases that describe depressive symptoms. The one-hot features were also used to train an LSTM-based deep RNN to represent and forecast unknown sensor text emotional states. Using the suggested method, the first and second datasets contain 11,807 and 21,807 texts, respectively. However, while mental characteristics appear to be the most important contributors to depression prediction, future analyses of these subsets in isolation and utilizing relevant data will enhance the classification performance and comprehension of the association between characteristics and depression. In the future, our method might be used to extract characteristics from social media, which is a current trend in ML methods. Classifying textual data in this way improves the ensemble system's reliability and sensitivity. Deep learning techniques like DNN might expand the ensemble classification range. As a result, this will be the subject of our next round of research to further refine this approach. Traditional techniques could only reach 91 percent mean recognition performance, suggesting the new approach's robustness. To create effective user interfaces for improved emotional care, the characteristics employed in this study can be leveraged to assist machine learning judgments. Deep learning with a large dataset may be an efficient system to be studied. Using cutting-edge technology, mental health services can assess and predict normal and severe mood problems in real-time.

## Figures and Tables

**Figure 1:** Sample post shows words belonging to the depression or nondepression category.

**Figure 2:** The proposed approach produces a fold-1 confusion matrix.

**Figure 3:** The proposed approach produces a fold-2 confusion matrix.

**Figure 4:** During trials on the dataset using the suggested technique, accuracy and loss of 10-folds were observed.

**Figure 5:** Traditional one-hot properties of two emotional states have been mapped out in a three-dimensional fashion by following LDA.

**Figure 6:** A 3-D representation of the typical TF-IDF properties of two emotional states is depicted following LDA.

**Figure 7:** Following PCA, shows a three-dimensional representation of the strong attributes predicted of two emotional states in three dimensions.

**Figure 8:** Emotional states are shown in a three-dimensional picture as a result of LDA.

**Algorithm 1:** Text feature extraction

**Algorithm 2:** A proposed model

**Table 1:** Words and phrases associated with depression are commonly used in English.

S.N.	Words
1	Nothing to eat
2	Ending my life is the only option I have left.
3	Suicide
4	Suicidal thoughts and tears
5	Take my own life away from me!
6	Take my life away from me.
7	a void of any kind
8	Sadness
9	Always drained in energy and lacking in inspiration
10	Not a thing
11	Nothing to do

LDA is used for a variety of purposes. To maximize interclass scatterings, LDA seeks to reduce scatterings inside a class.

**Table 2:** : Suicide and depression detection dataset Kaggle 233337 datasets.

Message	Case
Ex-wife threatening suicide recently I left my wife for good because she has cheated on me twice and lied to me so much that I have decided to refuse to go back to her. As of a few days ago, she began threatening suicide. I Have tirelessly spent these past few days talking her out of it and she keeps hesitating because she wants to believe I'll come back. I Know a lot of people will threaten this to get their way, but what happens if she does? What do I do and how am I supposed to handle her death on my hands? I Still love my wife but I cannot deal with getting cheated on again and constantly feeling insecure. I'm worried today may be the day she does it and I hope so much it does not happen.	Suicide
I Need help just help me I'm crying so hard	Suicide
It ends tonight. I Cannot do it anymore.	Suicide
Do you think getting hit by a train would be painful? Guns are hard to come by in my country but trains are not. I Just do not want to suffer through, do you think this would be a painless method of suicide?	Suicide
Iâ€™m scared. Everything just seems to be getting worse and worse. Iâ€™m young and I think Iâ€™m transgender but Iâ€™m not even sure about that. I canâ€™t tell if Iâ€™m just lying to myself or if Iâ€™m actually trans, I feel so overwhelmed with thoughts and emotions and I canâ€™t just take it anymore.	Suicide
I Just wish I could at least know for sure if I was trans, and even then I have to worry about if my (religious) family will be accepting and if I can do anything to alleviate my pain a bit.	
I Cut myself for the first time yesterday, I barely even drew blood so I canâ€™t even fucking hurt myself correctly. I donâ€™t think Iâ€™ll ever be able to do anything correctly, I want to pursue music but I know thereâ€™s no money to be found in that field unless I become famous but thatâ€™s not happening.	
Currently, Iâ€™m not seriously debating suicide but the thoughts keep coming back and they just keep getting worse. Iâ€™m is not sure if I can take this much longer, I just wish I was born a girl. I Want to cry.	
Am I weird I do not get affected by compliments if it's coming from someone I know IRL but I feel really good when Internet strangers do it	Nonsuicide
Everyone wants to be “edgy” and it's making me self-conscious I feel like I do not stand out. I Can draw yes and play the guitar but I honestly feel like being stuck in the past, my taste in music is all rock and alt-metal from 2000s to the ‘90s and it does not make me feel unique it's just my style but seeing as my friends and classmates get more into rap and EDM it's hard for me to feel like I fit in.	Nonsuicide
Then I do not feel like I stand out is because of all the others copying a style and if I do that I'd be just another	
“Quirky kid” who's in a cringe phase.	
Many of my friends say that I look good in grunge style and I kinda agree but it's hard for me to continue that if I cannot even stand out from all the “edgy	
People who wore crosses and wallet chains and do tiktoks”	
Feels like I do not fit in in all categories, am scared that people might confuse me with a CLOUT CHASER or a fucking TikTok *e* boy goddamn	
I Hate my life	
Hey, I'm gonna sleep with socks whatcha gonna do? Put them off?! good luck ima gonna sleep with warm feet	Nonsuicide

**Table 3:** For 100 epochs of training, the accuracy and loss are shown in a graph When a patient is suffering from depression.

State	Fold	Precision	Recall	F1-score	Support
Depression	1	0.95	0.97	0.96	189
	2	0.97	0.96	0.96	184
	3	0.96	0.94	0.95	187
	4	0.96	0.96	0.96	162
	5	0.99	0.94	0.97	190
	6	0.97	0.92	0.95	188
	7	0.95	0.99	0.97	172
	8	0.97	0.98	0.98	179
	9	0.97	0.98	0.98	179
	10	0.99	0.96	0.97	187

**Table 4:** 100 epochs of training in a nondepressive condition is shown to illustrate the accuracy and loss.

State	Fold	Precision	Recall	F1-score	Support
Nondepression	1	0.99	0.98	0.98	992
	2	0.98	0.99	0.98	997
	3	0.98	0.98	0.98	994
	4	0.99	0.99	0.99	1019
	5	0.98	0.99	0.99	991
	6	0.98	0.99	0.98	993
	7	0.99	0.98	0.99	1009
	8	0.99	0.99	0.99	1001
	9	0.99	0.99	0.99	1001
	10	0.98	0.99	0.99	993

**Table 5:** 100 epochs of training using the mean value as the state demonstrates the accuracy and loss during tenfold training.

State	Fold	Precision	Recall	F1-score	Support
Mean/Total	1	0.97	0.98	0.97	1181
	2	0.97	0.97	0.97	1181
	3	0.97	0.96	0.96	1181
	4	0.97	0.97	0.97	1181
	5	0.98	0.96	0.98	1181
	6	0.97	0.95	0.96	1181
	7	0.97	0.98	0.98	1181
	8	0.98	0.98	0.98	1181
	9	0.98	0.98	0.98	1181
	10	0.98	0.97	0.98	1181

**Table 6:** The accuracy of predictions made by various approaches for all people.

S.N.	Approaches	Mean accuracy (%)
1.	One-hot logistic regression	83.98
2.	Support vector machine	84.87
3.	Artificial neural network	83.56
4.	TF-IDF decision trees	82.25
5.	K-nearest neighbour	80.58
6.	Decision tree	84.25
7.	Ensemble model	87.69
8.	Usr2Vec	87.02
9.	MIL-SocNet	88.68
10.	TF-IDF deel model	88.26
11.	Proposed method	92.02

## Data Availability

The dataset has been downloaded from the website ung.no, which is a public Norwegian information website.
